This article has been retracted.

# Effects of Endoscopic Sinus Surgery Combined with Budesonide Treatment on Nasal Cavity Function and Serum Inflammatory Factors in Patients with Chronic Sinusitis

**DOI:** 10.1155/2022/4140682

**Published:** 2022-03-07

**Authors:** Yingying Zhao, Chenyan Jiang, Qingwei Wu, Runjie Shi

**Affiliations:** ^1^Department of Ortolaryngology, Huangpu Branch, Shanghai Ninth People's Hospital, Shanghai Jiao Tong University School of Medicine, Shanghai,200011, China; ^2^Department of Ortolaryngology, Shanghai Ninth People's Hospital, Shanghai Jiao Tong University School of Medicine, Shanghai 200011, China

## Abstract

In this article, we have explored the effects of endoscopic sinus surgery together with budesonide treatment on nasal function and serum inflammatory factors on patients with chronic sinusitis. We retrospectively analyzed 120 patients with chronic sinusitis who were admitted to our hospital from March 2018 to March 2021 and were eligible for this study. They were separated into 2 groups according to different treatments, that is, the control group (treated with endoscopic surgery alone) of 58 cases and observation group (treated with endoscopic sinus surgery combined with budesonide) with 62 cases. Treatment efficacy, surgical status, overall symptom score before and after treatment, nasal mucociliary clearance function, serum eosinophils (EOS), serum immunoglobulin E (IgE), serum inflammatory factors, and occurrence of adverse reactions of both groups were recorded and compared. Total effective rate in the observation group presented strikingly more positive compared with that among patients in control group (P<0.05), as well as the data recorded in terms of operation time, blood loss during surgery and postoperative improvement time of patients (P<0.05). Overall symptom score, nasal mucociliary clearance, EOS, IgE and serum inflammatory factors in both groups were improved notably after treatment, while the observation group held a more obvious improvement. And it also had a markedly lower incidence of adverse reaction (P<0.05). Endoscopic sinus surgery combined with budesonide in the treatment of chronic sinusitis could effectively improve the clinical symptoms of patients, reestablish the function of the nasal cavity and improve their inflammation level. Meanwhile, it was of high safety and is worthy of clinical promotion.

## 1. Introduction

Chronic sinusitis, one of the common diseases in otolaryngology, is characterized by multiple occurrence and recurrence. It is a disease in which non-specific infectious inflammation of the sinus mucosa and nasal cavity appears and lasts ≥ 12 weeks [1]. Chronic sinusitis is mainly caused by the involvement of multiple sinuses at one time, which will not only increase respiratory infections, but also cause other adverse reactions, such as cranio-ocular adverse reactions, affecting vision, and even aggravating infections, causing serious impacts on patients' health and quality of life and even death [2, 3].

With the advancement of minimally invasive surgery in recent years, endoscopic sinus surgery is often used in clinical practice to treat chronic sinusitis. It has the advantages of clear vision and easy lesion removal, and has been highly recognized by most patients and their families in clinical practice [4]. However, even if with endoscopic sinus surgery, it is still necessary to cooperate with drug treatment before and after surgery to reduce the tissue edema and inflammation of patients, lower the difficulty of endoscopic surgery, and decrease the recurrence rate of symptoms after surgery, which is of great help to control patient's condition [5, 6]. Relevant studies have shown that [7], on the basis of surgery, combined use of drugs for treatment can effectively improve the treatment effect. Inflammation is an important pathological basis for chronic sinusitis. The elevated levels of a variety of pro-inflammatory factors can accelerate the progression of the disease and aggravate the normal tissue damage of the nasal mucosa. Therefore, active anti-inflammatory treatment is also an important treatment for chronic sinusitis [8, 9]. Budesonide is a powerful anti-inflammatory and anti-allergic drug. After topical administration, it is beneficial to inhibit the activation of various inflammatory cells in the nasal cavity, reduce inflammatory damage in the lesion, and promote the absorption of mucosal edema, so as to accelerate the recovery of nasal function and relieve symptoms such as nasal congestion and purulent tears [10]. However, there are relatively few studies on the comprehensive efficacy of endoscopic sinus surgery combined with budesonide treatment in patients with sinusitis.

In this article, we have explored the effects of endoscopic sinus surgery together with budesonide treatment on nasal function and serum inflammatory factors on patients with chronic sinusitis. We retrospectively analyzed 120 patients with chronic sinusitis who were admitted to our hospital from March 2018 to March 2021 and were eligible for this study. They were separated into 2 groups according to different treatments, that is, the control group (treated with endoscopic surgery alone) of 58 cases and observation group (treated with endoscopic sinus surgery combined with budesonide) with 62 cases. Treatment efficacy, surgical status, overall symptom score before and after treatment, nasal mucociliary clearance function, serum eosinophils (EOS), serum immunoglobulin E (IgE), serum inflammatory factors, and occurrence of adverse reactions of both groups were recorded and compared.

The rest of the article is presented as given below.

In section 2, a detailed discussion on the effectiveness of the endoscopic sinus surgery together with budesonide treatment on nasal function and serum inflammatory factors on patients with chronic sinusitis is presented which is followed by a detailed discussion on the various experimental results and observations. These results were discussed and evaluated based on the problem at hand. Finally, concluding remarks are given to conclude the paper along with possible future directives and references which are used throughout the manuscript.

## 2. Proposed Mechanism or Evaluation Method

### 2.1. Clinical Information

We retrospectively analyzed 120 patients with chronic sinusitis who were admitted to our hospital from March 2018 to March 2021 and were eligible for this study, among which 64 cases were male and 56 cases were female. They were separated into 2 groups according to different treatments, that is, the control group (treated with endoscopic surgery alone) of 58 cases and observation group (treated with endoscopic sinus surgery combined with budesonide) with 62 cases.

#### 2.1.1. Inclusion Criteria

1. Included patients who meet the “Guidelines for the Diagnosis and Treatment of Chronic Rhinosinusitis”
2. Included patients with mucopurulent nasal discharge and nasal congestion
3. Included patients with nasal mucosal congestion, edema or polyps
4. Included patients who have been included in the course of disease for more than 1 year without obvious effects of drug treatment

#### 2.1.2. Exclusion Criteria:

1. Excluded patients with severe heart, lung, and renal insufficiency
2. Excluded patients with allergic rhinitis, nasal disease, etc.
3. Excluded patients allergic to glucocorticoids
4. Excluded patients with cystic fibrosis and congenital ciliary dyskinesia
5. Excluded patients with surgical intolerance
6. Excluded patients who do not cooperate with the study

All patients agreed to engage in present study with a informed consent form signed. And this experiment has been approved and accepted by the hospital ethics committee and also in conformity with the Helsinki Declaration.

### 2.2. Therapeutic Plan

Related preoperative examinations were perfected in both groups. The endoscopic sinus surgery was conducted in control group using Medtronic endoscopic sinus surgery system produced by Medtronic (USA). Patients were instructed to sit in the supine position. After successful anesthesia, the Messerklinger operation was selected to remove the uncinate process and open the maxillary sinus naturally. After the secretions and diseased tissues in the sinus cavity were completely removed, the anterior and posterior ethmoid sinuses were opened in an orderly manner, and then the diseased mucosa in the sinus cavity was removed. As the natural opening of the frontal sinus was enlarged and the diseased mucosa in the sinus cavity was removed, the ethmoid sphenoid plate was removed to open the sphenoid sinus. Lastly, the diseased tissue in the sinus cavity was properly removed. During the operation, mucosa should be restored as much as possible without destroying the normal structure. If the patient was accompanied by nasal polyps, surgeons should remove them and the stop the bleeding routinely after the operation. Patients in observation group started to use budesonide nasal spray (AstraZeneca Pharmaceutical Co., Ltd., National Medicine Standard: J201400483) nasal spray treatment 1 month before the operation. 2 sprays/time, 2 times/d at first use and then it was changed to 1 spray/time, 2 times/d. Both groups were followed up for 3 months.

### 2.3. Observation Index

1. Total effective rate of treatment of both groups were evaluated and compared. It was divided into markedly effective: patients who's symptoms disappeared, the sinus ostium recovered well, and the affected side had no thick secretions; effective: patients who's symptoms were relieved, and the affected side had mild edema accompanied by a small amount of secretion; invalid: patients who didn't reach up to above indicators. The total effective rate of treatment = (marked effective number + effective number)/total number x 100%.
2. operation time, surgical blood loss, and postoperative improvement time of both groups were recorded and compared. The shorter the time, the better the treatment.
3. Visual analogue scale (VAS) [11] was to evaluate the overall symptoms of both groups before and 4 weeks after the operation, including nasal congestion, runny nose, facial pain, hyposmia, etc. These symptoms are all represented by numbers from 0 to 10. 0 indicates asymptomatic, and 10 indicates the most severe symptoms;
4. Nasal mucociliary clearance function of two groups of patients were evaluated by the saccharin experiment, including mucociliary clearance speed, saccharin clearance time, and nasal mucociliary clearance rate.
5. The automatic blood cell analyzer (XFA6100, Beijing Pulang New Technology Co., Ltd.) was utilized to detect the serum eosinophils (EOS) of both groups before and after treatment; the enzyme-linked immunosorbent assay (ELISA) was applied to detect serum immunoglobulin E (IgE) of patients before and after treatment.
6. ELISA method was utilized for detection of serum inflammatory factors, including levels of tumor necrosis factor-*α* (TNF-*α*), interleukin-6 (IL-6) and interleukin-8 (IL-8) before and after treatment.
7. The occurrence of adverse reactions of both groups were recorded and compared, which included nasal cavity adhesion, epistaxis, sinus orifice blockage, and tear duct damage.

### 2.4. Statistical Methods

In present study, SPSS 19.0 statistical software was applied for statistical analysis of the data collected, GraphPad 8 for pictures required, percentage (%) for data counting, chi-square test for statistic analysis, independent t test for comparison of measured data, paired t test for comparison before and after treatment, and P<0.05 indicated the difference was of statistical significance.

## 3. Experimental Results and Evaluations

### 3.1. General Information Comparison

Two groups of patients were comparable due to negligible differences in gender, age, smoking history, etc. (P>0.05).  Table 1.

### 3.2. Comparison of the Therapeutic Effect of Both Groups

Patients were evaluated after treatment, and the number of patients who were markedly effective, effective and invalid in the observation group was 35, 25, and 2 respectively, with an effective rate of 96.15%. And those in the control group was 27, 20 and 11 respectively, and the treatment effective rate was 79.17%, indicating that observation group had a notably better therapeutic efficiency (P<0.05).  Table 2.

### 3.3. Comparison of operation duration, surgery blood loss, and postoperative improvement time between groups

The length of operation, the amount of blood loss and the time of postoperative improvement of observation group were notably shorter compared with control group, (P<0.05). Details were shown in Table 3.

### 3.4. Comparison of the symptom VAS scores in two groups before and after surgery

No striking difference presented in terms of overall symptom VAS scores between two groups before surgery (P>0.05); while it went significantly lower in both groups 4 weeks after surgery (P<0.05), and observation group had a more marked decrease comparatively (P<0.05).  Table 4.

### 3.5. Comparison of nasal mucociliary clearance before and after treatment between two groups

No marked distinction presented regarding nasal mucociliary function between two groups before surgery (P>0.05); while it was markedly improved in both groups after intervention (P<0.05), and observation group held a comparatively higher clearance rate of mucociliary and shorter clearance time of saccharin (P<0.05).  Figure 1.

### 3.6. Comparison of Serum EOS and Ige of Two Groups before and After Surgery

No marked distinction shown regarding serum IgE and EOS levels in two groups before treatment (P>0.05); while after treatment, the serum IgE and EOS levels in the control group were (63.93±2.70) kU/L and (3.94±0.36) % respectively. And those in observation group were (55.23±2.11) kU/L and (3.02±0.25)%, respectively, which were both drastically lower than before (P<0.05); among which, that in observation group went lower comparatively in the same period (P<0.05), Figure 2.

### 3.7. Comparison of serum inflammatory factors before and after operation between two groups

No notable distinct presented regarding inflammatory factors levels between two groups before treatment (P>0.05); after treatment, the levels of serum TNF-*α*, IL-8 and IL-6 in both groups went drastically lower, and the decrease in observation group was more notable when it was compared with control group (P<0.05).  Figure 3.

### 3.8. Comparison of the incidence of adverse reactions between groups after surgery

Patients' adverse reactions were recorded and compared after treatment. The number of patients in the observation group who had nasal cavity adhesions, epistaxis, sinus orifice blockage, and tear duct injury were 1, 2, 1, and 1, respectively, with an incidence of adverse reactions of 8.06%. While when it comes to control group, the numbers of which were 4, 4, 3, and 2, respectively, showing an incidence of adverse reactions of 22.41%, which was strikingly higher than that in observation group (P<0.05).  Table 5.

## 4. Discussion

Chronic sinusitis is a disease characterized by cavity inflammation, with main symptoms of nasal congestion, sticky or purulent discharge, and headache. If not treated in time, it will affect patient's eye nerves and functions, resulting in adverse reactions such as vision loss. It can also cause intracranial infection, causing headaches, fever, vomiting and other symptoms, severely impairing patient's physical function and bringing serious impact and damage to patient's normal life [12, 13]. The incidence of chronic sinusitis is relatively high. Thus, in the clinical treatment of this disease, nasal endoscopic surgery is often used as the local anatomical structure can be clearly observed, meanwhile, the diseased tissue can be understood and targeted in time to effectively restore the basic functions of the sinuses and nasal cavity [14]. Although nasal endoscopic surgery could effectively improve the therapeutic effect, it will inevitably increase the secretion of inflammatory mediators due to invasive operations. Therefore, it is of necessity to apply drugs on the basis of surgical treatment to improve clinical efficacy [15]. For further exploration of the appropriate treatment options for chronic sinusitis patients, we analyzed the therapeutic effect of endoscopic sinus surgery combined with budesonide in patients with chronic sinusitis.

We first compared the treatment efficacy of two groups of patients, and it showed that the treatment efficacy of the observation group was notably better, and the operation time, surgical blood loss, and postoperative improvement time of the observation group were strikingly less comparatively. This suggested that the use of budesonide before surgery was beneficial for surgical efficacy and the implementation of surgery. The main component of budesonide suspension is glucocorticoid, which has a definite anti-inflammatory effect and can inhibit the activation of macrophages, eosinophils and neutrophils. Administration through nasal aerosol inhalation helps to promote the direct action of the drug on the local nasal cavity and sinus mucosa, thereby facilitating the full absorption of the drug in the mucosa and enhancing the pharmacological effect of the drug [16, 17]. The results of this study suggested that endoscopic sinus surgery combined with budesonide could help reduce surgical damage and shorten the recovery time of chronic sinusitis patients. Immediately afterwards, we compared the symptom scores and nasal mucociliary clearance function of two groups before and after surgery, indicating that the VAS score and nasal mucociliary clearance function of both groups were markedly improved after treatment, and the improvement of observation group is comparatively more obvious. Nasal mucosal cilia system is mainly composed of cilia, glands, periciliary fluid, secretory cells, etc., which is particularly important for preventing the invasion of pathogenic bacteria and reducing the occurrence of infectious diseases [18]. Result of this indicator suggested that endoscopic sinus surgery combined with budesonide could better improve patient's symptoms and restore their nasal mucociliary clearance function.

Subsequently, we compared the expressions of serum EOS, IgE, IL-6, IL-8, and TNF-*α* in two groups. Results suggested that the EOS, IgE, and IL-6, IL-8, and TNF- *α* were effectively improved, and the improvement of observation group is markedly obvious. Former studies have suggested that EOS would increase in patients with chronic sinusitis and gradually accumulate in the lesions of the nasal mucosa, thereby aggravating the lesions [19]. IgE is human immunoglobulin E, which is produced when the body is stimulated [20], and it has been clinically proven that the serum levels of EOS and IgE in patients with chronic sinusitis will significantly increase [12]. IL-6 is mainly secreted by B cells, T cells, etc., and can form an inflammation cascade network with TNF-*α*, plays an important role in the body's anti-infection immunity, and can inhibit the immune function of CRS patients [21]. TNF-*α* can initiate and promote a variety of inflammatory reactions, and IL-8 has a chemotactic effect and induces the aggregation of inflammatory factors [22, 23]. Previous studies have reported that the serum inflammatory factor levels of patients with chronic sinusitis were higher compared with healthy people, which was not conducive to the treatment of chronic sinusitis. Therefore, it is very important to decrease the level of peripheral blood inflammatory factors of patients with chronic sinusitis [24]. This study showed that after treatment, the levels of IgE and EOS in both groups were significantly reduced, and the decline in the observation group was notably greater compared with the control group. And the levels of inflammatory factors presented similar changes as the igE and EOS level, both declined after intervention and observation group held better improvent. After analysis of the reasons, we believe that budesonide, as a glucocorticoid, had a local anti-inflammatory effect and could alleviate the inflammatory response in patients with chronic sinusitis and reduce the level of inflammatory factors [25]. And budesonide could also reduce the contraction response of smooth muscles, enhance the stability of endothelial cells and lysosomal membranes, alleviate the clinical symptoms of chronic sinusitis, and reduce IgE and EOS levels [26]. Finally, to evaluate the safety of the combined treatment plan, we took notes on the incidence of adverse reactions in both groups. Results revealed that the observation group had a strikingly lower incidence of adverse reactions, indicating that endoscopic sinus surgery combined with budesonide in the treatment of chronic sinusitis could better reduce the occurrence of adverse reactions and has better safety.

## 5. Conclusion

In this article, we have explored the effects of endoscopic sinus surgery together with budesonide treatment on nasal function and serum inflammatory factors on patients with chronic sinusitis. We retrospectively analyzed 120 patients with chronic sinusitis who were admitted to our hospital from March 2018 to March 2021 and were eligible for this study. They were separated into 2 groups according to different treatments, that is, the control group (treated with endoscopic surgery alone) of 58 cases and observation group (treated with endoscopic sinus surgery combined with budesonide) with 62 cases. Treatment efficacy, surgical status, overall symptom score before and after treatment, nasal mucociliary clearance function, serum eosinophils (EOS), serum immunoglobulin E (IgE), serum inflammatory factors, and occurrence of adverse reactions of both groups were recorded and compared. Finally, the combination of endoscopic sinus surgery and budesonide in chronic sinusitis treatment could effectively improve patients' clinical symptoms, restore the nasal cavity function and improve the level of inflammation. Moreover, it was of high safety and is worthy of clinical promotion.

## Figures and Tables

**Figure 1:** Comparison of nasal mucociliary clearance before and after treatment between two groups of patients; (a) comparison of mucociliary clearance of two groups before and after treatment; (b) comparison of saccharin clearance time between two groups of patients before and after treatment; (c) comparison of mucociliary clearance rate in two groups of patients before and after treatment.^∗^*P*<0.05.

**Figure 2:** Comparison of serum EOS and Ige between two groups of patients before and after surgery; (a) comparison of serum EOS and IgE between two groups of patients before and after treatment; (b) comparison of serum IgE between two groups of patients before and after treatment. ^∗^*P*<0.05.

**Figure 3:** Comparison of serum inflammatory factors before and after operation of two groups; (a) comparison of the serum IL-6 of two groups before and after the operation; (b) comparison of serum IL-8 of two groups before and after the operation; (c) comparison of serum TNF-*α*between two groups of patients before and after surgery.^∗^*P*<0.05.

**Table 1:** General information table (*n* (%)).

Factors	Observation group *n* = 62	Control group *n* = 58	*t/X2*	*P*
Gender			0.134	0.715
Male	32 (51.61)	28 (48.28)		
Female	30 (48.39)	30 (51.72)		
Age (years)			0.001	0.981
≤37	33 (53.23)	31 (53.45)		
>37	29 (46.77)	27 (46.55)		
BMI(kg/m2)			0.046	0.831
≤23	33 (53.23)	32 (55.17)		
>23	29 (46.77)	26 (44.83)		
History of smoking			0.013	0.909
YES	40 (64.52)	38 (65.52)		
NO	22 (36.48)	20 (34.48)		
Course of disease (years)			1.505	0.220
≤2	27 (43.55)	25 (55.56)		
>2	35 (56.45)	33 (44.44)		
Clinical classification			0.073	0.964
Type I	22 (35.48)	20 (34.48)		
Type II	21 (33.87)	21 (36.21)		
Type III	19 (30.65)	17 (29.31)		

**Table 2:** Comparison of therapeutic effects between the two groups of patients

Therapeutic efficiency	Observation group *n* = 62	Control group *n* = 58	t	P
Markedly Effective	35(56.46)	27(46.55)	-	-
Effective	25(40.32)	20(34.48)	-	-
Invalid	2(3.23)	11(18.97)	-	-
Effective rate	60(96.77)	47(81.83)	7.685	0.006

**Table 3:** Comparison of operation time, operation blood loss, and postoperative improvement time of two groups of patients.

Surgical situation	Observation group *n* = 62	Control group *n* = 58	t	P
Operation duration (min)	46.48±2.09	63.11±3.11	34.58	<0.001
Surgery blood loss (ml)	75.24±3.74	92.96±2.68	29.65	<0.001
Postoperative improvement time (d)	5.21±0.64	6.47±0.74	9.99	<0.001

**Table 4:** Comparison of the symptom VAS scores of two groups before and after surgery.

When	Observation group *n* = 62	Control group *n* = 58	t	P
Before operation	20.67 ± 2.26	20.96 ± 2.77	0.630	0.530
After operation	5.11 ± 0.68	6.55 ± 0.72	11.27	<0.001

**Table 5:** Comparison of the incidence of adverse reactions between two groups after surgery.

Adverse reactions	Observation group *n* = 62	Control group *n* = 58	T	P
Nasal cavity adhesions	1(1.61)	4(6.90)	-	-
Epistaxise	2(3.23)	4(6.90)	-	-
Sinus orifice blockage	1(1.61)	3(5.17)	-	-
Tear duct injury	1(1.61)	2(3.45)	-	-
Incidence of adverse reactions	5(8.06)	13(22.41)	4.839	0.028

## Data Availability

The simulation experiment data used to support the findings of this study are available from the corresponding author upon request.

## References

[1] Zheng L., Feng H., Yin L. (2021). Study on the correlation factors of tumour prognosis after intravascular interventional therapy. *Journal of Healthcare Engineering*.

[2] Ghogomu N., Kern R. (2017). Chronic rhinosinusitis: the rationale for current treatments. *Expert Review of Clinical Immunology*.

[3] Shetty K. R., Soh H. H., Kahn C. (2020). Review and analysis of Research trends in surgical treatment of pediatric chronic sinusitis. *American Journal of Rhinology & Allergy*.

[4] Kern R. C., Stolovitzky J. P., Silvers S. L. (2018). A phase 3 trial of mometasone furoate sinus implants for chronic sinusitis with recurrent nasal polyps. *International Forum of Allergy & Rhinology*.

[5] Ramakrishnan V. R. (2019). Ergonomics in endoscopic sinus surgery. *Current Opinion in Otolaryngology & Head and Neck Surgery*.

[6] Sowerby L. J., Harris M. S., Joshi R., Johnson M., Jenkyn T., Moore C. C. (2020). Does endoscopic sinus surgery alter the biomechanics of the orbit?. *Journal of Otolaryngology - Head & Neck Surgery*.

[7] Amorocho M. C., Fat I. (2016). Anesthetic techniques in endoscopic sinus and skull base surgery. *Otolaryngologic Clinics of North America*.

[8] Ginat D. T. (2015). Posttreatment imaging of the paranasal sinuses following endoscopic sinus surgery. *Neuroimaging Clinics of North America*.

[9] Siu J., Shrestha K., Inthavong K., Shang Y., Douglas R. (2020). Particle deposition in the paranasal sinuses following endoscopic sinus surgery. *Computers in Biology and Medicine*.

[10] Thanneru M., Lanke S., Kolavali S. (2020). The effectiveness of budesonide nasal irrigation after endoscopic sinus surgery in chronic allergic rhinosinusitis with polyps. *Indian Journal of Otolaryngology and Head & Neck Surgery*.

[11] Chen F.-H., Deng J., Hong H.-Y. (2016). Extensive versus functional endoscopic sinus surgery for chronic rhinosinusitis with nasal polyps and asthma: a 1-year study. *American Journal of Rhinology & Allergy*.

[12] Alsaleh S., Manji J., Javer A. (2019). Optimization of the surgical field in endoscopic sinus surgery: an evidence-based approach. *Current Allergy and Asthma Reports*.

[13] Tsuzuki K., Hashimoto K., Okazaki K., Sakagami M. (2018). Post-operative course prediction during endoscopic sinus surgery in patients with chronic rhinosinusitis. *Journal of Laryngology & Otology*.

[14] Richards J. P., Done A. J., Barber S. R., Jain S., Son Y. J., Chang E. H. (2020). Virtual coach: the next tool in functional endoscopic sinus surgery education. *International Forum of Allergy & Rhinology*.

[15] Fortes B., Balsalobre L., Weber R. (2016). Endoscopic sinus surgery dissection courses using a real simulator: the benefits of this training. *Brazilian Journal of Otorhinolaryngology*.

[16] Soudry E., Wang J., Vaezeafshar R., Katznelson L., Hwang P. H. (2016). Safety analysis of long-term budesonide nasal irrigations in patients with chronic rhinosinusitis post endoscopic sinus surgery. *International Forum of Allergy & Rhinology*.

[17] Kang T. W., Chung J. H., Cho S. H., Lee S. H., Kim K. R., Jeong J. H. (2017). The effectiveness of budesonide nasal irrigation after endoscopic sinus surgery in chronic rhinosinusitis with asthma. *Clinical and Experimental Otorhinolaryngology*.

[18] Liu Y., Zhang Z. Y. (2016). Effects of staphylococcus aureus hemolysin on nasal mucociliary clearance system. *Lin Chung Er Bi Yan Hou Tou Jing Wai Ke Za Zhi*.

[19] Shi Y., Ji R., Zhang G., Wang W., Lin P. (2021). The influence of contoured sinus endoscopy on the recurrence of nasal polyps. *Lin Chung Er Bi Yan Hou Tou Jing Wai Ke Za Zhi*.

[20] Lal D., Baroody F. M., Weitzel E. K., deTineo M., Naclerio R. M. (2006). Total IgE levels do not change 1 year after endoscopic sinus surgery in patients with chronic rhinosinusitis. *International Archives of Allergy and Immunology*.

[21] Van Zele T., Holtappels G., Gevaert P., Bachert C. (2014). Differences in initial immunoprofiles between recurrent and nonrecurrent chronic rhinosinusitis with nasal polyps. *American Journal of Rhinology & Allergy*.

[22] Wei L., Zhang Y., Tan H. (2018). Changes of TNF-伪, PDGF and HA in nasal secretions and olfactory function of patients with chronic sinusitis before and after endoscopic sinus surgery. *Experimental and Therapeutic Medicine*.

[23] Wang C. S., Honeybrook A., Chapurin N., Keswani A., Jang D. W. (2017). Sinusitis in patients on tumor necrosis factor alpha inhibitors. *International Forum of Allergy & Rhinology*.

[24] Ma M., Liu L., Jin W., Chen H., Zhou T., Tong B. (2021). Study on the effects of desloratadine citrate disodium on the postoperative complications and inflammatory response in patients with chronic sinusitis undergoing endoscopic sinus surgery. *American Journal of Tourism Research*.

[25] Huang Z.-z., Chen X.-z., Huang J.-c. (2019). Budesonide nasal irrigation improved Lund-Kennedy endoscopic score of chronic rhinosinusitis patients after endoscopic sinus surgery. *European Archives of Oto-Rhino-Laryngology*.

[26] Zhang L. W., Reng M. X., Xue G. C. (2016). Astragalus granule combined auricular point sticking for cough variant asthma in children. *Zhongguo Zhong Xi Yi Jie He Za Zhi*.

